The article "Care Bundles plus Detailed Nursing on Mortality and Nursing Satisfaction of Patients with Septic Shock in ICU" was retracted in 2023. Reasons: unreliable results or conclusions; concerns about the data; concerns about the peer review; concerns about the citations.

# Care Bundles plus Detailed Nursing on Mortality and Nursing Satisfaction of Patients with Septic Shock in ICU

**DOI:** 10.1155/2022/1177961

**Published:** 2022-06-23

**Authors:** Min Wang, Yan Zhang, Ailing Zhong, Fen Zhou, Haibo Wang

**Affiliations:** Department of Critical Care Medicine, Hai'an People's Hospital, Nantong, Jiangsu 226600, China

## Abstract

**Objective:**

To evaluate the effect of care bundles combined with detailed nursing on the mortality and nursing satisfaction of patients with septic shock in the intensive care unit (ICU).

**Methods:**

Ninety patients with septic shock in the ICU admitted to our hospital from April 2019 to April 2020 were recruited and assigned to an experimental group and a control group via the random table method, with 45 cases in each group. The control group adopted conventional nursing, and the experimental group received care bundles combined with detailed nursing. The nursing effect, satisfaction, and mortality of the two groups were compared. The “Glasgow Coma Scale” (GCS) was used to evaluate the coma of the patients, the “Coma Recovery Scale” (CRS-R) was used to assess the state of consciousness of the patients, and the “Hospital Anxiety and Depression” (HAD) scale was used to evaluate the patient's emotional status before and after the intervention.

**Results:**

The experimental group showed a significantly higher nursing efficiency and better nursing satisfaction than the control group (*P* < 0.05). Lower mortality was found in the experimental group in contrast to the control group (*P* < 0.05). The experimental group had higher GCS scores and CRS-R scores and lower HAD scores than the control group (*P* < 0.05).

**Conclusion:**

Care bundles plus detailed nursing for patients with septic shock in the ICU improve the nursing effect and nursing satisfaction, reduce the mortality rate, and mitigate the clinical symptoms of patients, which shows great potential in clinical application and promotion.

## 1. Introduction

Septic shock is a serious clinical syndrome caused by Gram-negative bacterial infections and triggers microcirculation disorders and compromises blood perfusion in different tissues, resulting in inflammation and organ disorders, with extremely high mortality. The delay of treatment may be life-threatening to the patients [1–3]. Sepsis is a critical disease with a poor prognosis, and infection is the common cause. Infections compromise the oxygen metabolism of the organism, decrease oxygen utilization, activate inflammatory responses, and cause mitochondrial dysfunction, thereby triggering hypoxia in the organism [4]. Moreover, in the presence of infection, vasodilation and increased vascular permeability cause tissue edema, and insufficient circulating blood volume leads to inadequate tissue perfusion and decreased blood circulation [5]. The susceptible populations for sepsis include those who are immunocompromised, malignant, aging, and overmedicated. Nursing care of patients with infectious shock in the intensive care unit (ICU) requires systematic, comprehensive, and integrated nursing interventions, close monitoring of patients' vital signs, and improved safety and standardized management, including infusion control, medication guidance, and abnormal emotional mitigation. Care bundles have emerged in recent years as a new type of nursing that provides patients with more comfort in nursing and promotes patient recovery, with an increase of 50% in the nursing efficiency [4–6]. Care bundles combined with detailed nursing provide patients with better medical services and improve the quality of care and the prognosis of patients. In traditional Chinese medicine (TCM), sepsis is classified as an “external febrile disease,” and the basic pathogenesis of sepsis is deficiency, toxicity, stasis, and blood stagnation [7, 8]. TCM treatment for sepsis follows the principle of benefiting qi and nourishing yin, clearing heat and detoxifying toxins, activating blood circulation, and resolving blood stasis. It has been shown that TCM adjuvant therapy improves the prognosis of patients with sepsis [7, 8], but TCM combined with care bundles plus detailed nursing has been rarely reported. Therefore, the present study innovatively incorporates TCM treatment with quality nursing intervention for sepsis patients. The report is as follows.

## 2. Materials and Methods

### 2.1. Ethical Statement

The study was approved by the Hospital Ethics Committee, and the patients and their families were informed of the purpose and process of the study and signed the informed consent.

### 2.2. General Information

A total of ninety patients with septic shock in the ICU admitted to our hospital from April 2019 to April 2020 were selected as the research objects and assigned to an experimental group and a control group via the random table method, with 45 cases in each group. Inclusion criteria: all patients who met the sepsis-3 sepsis diagnostic criteria as revised in the 2016 edition of the conference on the Definition of Septic Shock and Sepsis in Europe and the United States [4] and with no history of coagulopathy or severe organ failure were included. Exclusion criteria: patients with severe hepatic and renal dysfunction, autoimmune diseases, and psychiatric disorders, during pregnancy or lactation, in a terminal state, and with severe renal dysfunction were excluded.

### 2.3. Method

All patients were treated with anti-infective treatment after admission, and treatment measures such as cardiac function strengthening, blood volume supplement, cerebral edema prevention, acidosis correction, antiplatelet aggregation, and microcirculation improvement were adopted [7].

The patients in the control group received routine nursing, including real-time monitoring of the vital signs, respiratory tract nursing, medication instruction, and close observation of the changes in the patient's condition.

The experimental group adopted care bundles combined with detailed nursing. (1) Establishment of a nursing team, with the head nurse of the ICU as the team leader and the responsible nurses of the ICU as the team members. Medical staff received care bundle training regularly to deepen their understanding of the nursing model. Members of the team were required to retrospectively analyze issues and care risks that may occur in the nursing process and formulate corresponding solutions. The detection of the patients' vital signs was as follows: blood pressure of the patients was measured every 15 min, and rectal temperature was measured every 120 min with their central venous pressure stabilized between 60 and 110 mm H_2_O, arterial pressure maintained above 64 mm·Hg, and blood oxygen saturation maintained above 92% [8]. The changes in the patient's blood glucose level were determined. The patient's blood glucose level was maintained below 8.5 mmol/L. The patient's daily fluid intake and output were also recorded. (2) Medication nursing. Before pathogen culture and drug susceptibility testing, the patients were first treated with broad-spectrum antibiotics. The patient's hematocrit was maintained at over 33%, and an infusion of concentrated red blood cells was performed when the hemoglobin level was reduced to under 73 g/L. The patients were promptly given alkaline drugs in the event of acidosis [9]. The use of vasoactive drugs required close attention to the patient's blood pressure and heart rate. (3) Patients with breathing difficulties or respiratory depression were given oxygen therapy. Changes in the patient's vital signs during oxygen therapy were monitored. The secretions in the patient's mouth and nose were timely cleaned up to ensure smooth breathing. Intubation and mechanical ventilation were applied if necessary. (4) Safety management. Patients with septic shock may suffer agitation, which requires proper safety management [10]. For patients with limb tremors, a restraint belt was used to restrain their movement. All tubes were properly handled to prevent from twisting, bending, and dropping out. (5) Nutrition support. Nasogastric tubes were indwelled for infusing enteral nutrition to the patients, with careful control of the infusion dose and infusion speed to avoid gastric retention, during which the bed was raised to avoid gastric reflux. The temperature of the nutrient was maintained at 38–40°C. (6) Anti-infective and symptomatic treatment. Vasoactive drugs were used to maintain the patients' blood pressure, and the corresponding drugs were used for the infected lesion. The patient's medication, vital signs, and organ tissue perfusion were closely monitored [11]. (7) Preventive nursing for complications. The patients' catheters and urine bags were replaced in time, and their perineum was cleaned daily to avoid infection of the urinary system. Sputum suction care was conducted to prevent the occurrence of pneumonia. (9) Psychological nursing. The patients' mental states were closely monitored to timely relieve their negative emotions, reduce the psychological pressure, and ensure a high degree of treatment cooperation [12].

All patients received Fusu Pills for TCM adjuvant therapy. The ingredients of the pills include Panax quinquefolius, Astragali Radix, raw Rhei Radix et Rhizoma, raw Gypsum Fibrosum, Ophiopogonis Radix, Salviae Miltiorrhizae Radix et Rhizoma, Paeoniae Radix Rubra. The above herbs were ground and packed into capsules (0.4 g per capsule). The patients received 4 capsules through oral or nasal administration thrice daily.

### 2.4. Observational Indexes

The nursing effect of the two groups of patients was evaluated with reference to the International Guidelines for the Treatment of Severe Sepsis and Septic Shock [13]. Significantly effective: after the nursing, the patients had mitigated clinical symptoms and restored consciousness without complications. Effective: after the nursing, the patients had relieved clinical symptoms and restored consciousness with minor complications. Ineffective: after the nursing, the clinical symptoms and consciousness showed no changes, with serious complications (number of significantly effective cases + number of effective cases)/total number of cases *∗* 100% = total efficiency.

The “Patient Clinical Satisfaction Questionnaire” prepared by the department was used to investigate the satisfaction of patients after nursing. The total score on the scale is 100 points. The higher the score, the higher the patient satisfaction.

The “Glasgow Coma Scale” [13] (GCS) was used to assess the degree of coma of the patients. The scale mainly includes verbal response, limb response, and eye-opening response. The score was adversely proportional to the severity of the coma.

The “Coma Recovery Scale” [14] (CRS-R) was used to evaluate the state of consciousness of the patients, and the score was proportional to the state of consciousness.

The Hospital Anxiety and Depression Scale [15] (HAD) was used to assess the emotional state of patients before and after the intervention, with a total score of 42 points. The higher the score, the more severe the anxiety and depression of the patient.

### 2.5. Statistical Processing

SPSS20.0 was used for data analysis, and GraphPad Prism 7 (GraphPad Software, San Diego, USA) was employed to plot the graphics. The research included count data and measurement data. The count data were analyzed by the chi-square test, and the measurement data were analyzed by the *t*-test and normal distribution. *P* < 0.05 indicates statistical significance.

## 3. Results

### 3.1. General Information

The two groups showed no great disparity in age, gender, BMI, smoking, drinking, and the place of residence (*P* > 0.05), as shown in Table 1.

### 3.2. Nursing Satisfaction

In the experimental group, there were 32 (71.11%) cases of satisfied, 10 (22.22%) cases of moderately satisfied, and 3 (6.67%) cases of dissatisfied, with an overall satisfaction rate of 93.33%. In the control group, there were 20 (44.44%) cases of satisfied, 13 (28.89%) cases of moderately satisfied, and 12 (26.67%) cases of dissatisfied, with an overall satisfaction rate of 73.33%. Patients in the experimental group were more satisfied with the nursing versus those in the control group (*X*^2^ = 6.480, *P* < 0.05) (Figure 1).

### 3.3. Nursing Effects

In the experimental group, there were 26 (57.78%) significantly effective cases, 16 (35.56%) effective cases, and 3 (6.67%) ineffective cases. In the control group, there were 21 (46.67%) significantly effective cases, 10 (22.22%) effective cases, and 14 (31.11%) ineffective cases. The total efficiency of the experimental group (93.33%) was higher than that of the control group (68.89%) (*X*^2^ = 8.775, *P* < 0.05), as shown in Table 2.

### 3.4. GCS Score

Before the intervention, the limb response, eye-opening response, and verbal response were 2.31 ± 0.47, 1.96 ± 0.24, and 2.23 ± 0.76 in the experimental group and 2.46 ± 0.42, 1.83 ± 0.37, and 2.29 ± 0.77 in the control group. After the intervention, the limb response, eye-opening response, and verbal response were 4.73 ± 1.12, 4.73 ± 1.12, and 4.73 ± 1.12 in the experimental group and 3.17 ± 0.93, 2.18 ± 0.54, and 3.12 ± 0.47 in the control group. The GCS scores in the experimental group were significantly higher than those of the control group (*P* < 0.05) (Table 3).

### 3.5. CRS-R Score

The CRS-R scores of the patients in the experimental group before and after intervention were 3.54 ± 1.17 points and 20.25 ± 1.37 points, respectively.

The CRS-R scores of the control group before and after intervention were 3.59 ± 1.18 points and 17.14 ± 1.26 points, respectively. After treatment, the CRS-R scores of the two groups were significantly increased, with higher results in the experimental group (*P* < 0.05) (Figure 2).

### 3.6. HAD Score

The HAD scores of the patients in the experimental group before and after the intervention were 35.81 ± 3.25 points and 5.36 ± 1.21 points, respectively. The HAD scores of the patients in the control group before and after the intervention were 35.88 ± 3.22 points and 13.29 ± 2.53 points, respectively. After treatment, the HAD scores of the two groups were significantly reduced, with lower results in the experimental group (*P* < 0.05) (Figure 3).

### 3.7. Mortality Rate

No death records were obtained in the experimental group, and a total of 5 cases of death were recorded in the control group with a mortality rate of 12.5%. The mortality rate of the experimental group was significantly lower than that of the control group (*P* < 0.05).

## 4. Discussion

Septic shock is a common critical illness caused by the invasion of viruses and microorganisms in the circulatory system. ICU patients are critically ill, with poor physical fitness and low immunity. Moreover, the intubation of various tubes such as tracheal tubes, gastric tubes, central venous catheters, and urinary catheters predisposes the patients to multiple infections. After the onset of septic shock, patients are prone to a decrease in microcirculation perfusion of body tissues, followed by impaired organ function, hypoxia in tissues and systems, and even organ failure, which can be life-threatening to the patients [16–19]. Currently, ulinastatin and low molecular heparin, antiinfective treatment, symptomatic treatment, and the maintenance of water-electrolyte balance and acid-base balance are mainly used in clinical practice to maintain the patient's vital signs and improve patients' acute physiological and chronic health status scores and Marshall scores, clinical outcomes, and inflammatory factors such as serum tumor necrosis factor-alpha, interleukin-6, and interleukin-8.

Care bundles are targeted nursing measures tailed for each patient based on their actual conditions [20–22]. The combination of care bundles with detailed nursing requires proper medication, close monitoring of patients' vital signs, oxygen inhalation nursing, nutritional care, safety management, and active communication with the patients, so as to alleviate the patients' clinical symptoms, get control of the disease condition, mitigate the patients' negative emotions and psychological pressure, and build up confidence in treatment, which contributes to the enhancement of treatment compliance and the acceleration of patients' recovery [23]. The results of this study showed that the total nursing efficiency of patients in the experimental group was significantly higher than that of the control group (*P* < 0.05), which was consistent with the research results of PHILLIPS [24] et al. In their research, they used developmental scales to quantify and improve acuity of care, predict patient prognosis, length of stay and resource utilization, and improve the treatment efficiency, in which “the total effective rate of the observation group was 95.3%, significantly higher than the total effective rate of 87.6% in the control group (*P* < 0.05).” It proves that care bundles combined with detailed nursing could effectively improve the efficiency of nursing, abate the clinical symptoms of patients, and reduce the mortality rate of patients.

Following the release of the international guidelines for the treatment of severe sepsis and septic shock [10, 11], the morbidity and mortality rate of severe sepsis have shown a year-on-year decrease. The improvement of adherence to this guideline is an important measure to promote its promotion and improve the prognosis of patients with severe sepsis [12]. The absence of improvement in morbidity and mortality is associated with the lack of strict compliance with physician guidelines by nursing staff or inefficient information transfer in shift exchange [13]. Care bundles combined with detailed nursing used in the present study improve medical advice compliance, multidisciplinary cooperation, and ICU resource rationing, thereby increasing the treatment efficiency of sepsis. Due to the complex pathological mechanisms of sepsis, drug resistance may easily occur during treatment [14]. Thus, future in vitro studies on the pathological mechanisms of sepsis and screening of drug targets for molecular mechanisms such as signaling pathways are required to obtain better clinical efficacy.

## 5. Conclusion

Care bundles plus detailed nursing for patients with septic shock in ICU improve the nursing effect and nursing satisfaction, reduce the mortality rate, and mitigate the clinical symptoms of patients, which shows great potential in clinical application and promotion. The limitation of this study is the potential bias due to the small sample size and lack of evidence-based translational studies, which requires further incorporation of evidence-based evidence. In addition, there is no long-term follow-up data of patients in this study, so long-term follow-up will be conducted in future studies to obtain more reliable data.

## Figures and Tables

**Figure 1:** Comparison of satisfaction between the two groups [*n *(%)]. Note: Figure (a) is the nursing satisfaction results of the experimental group; Figure (b) is the nursing satisfaction results of the control group; the satisfied rate of the experimental group was 71.11% (32/45), the moderately satisfied rate was 22.22% (10/45), the dissatisfied rate was 6.67% (3/45), and the overall satisfaction rate was 93.33% (42/45); the satisfied rate of the experimental group was 44.44% (20/45), the moderately satisfied rate was 28.89% (13/45), the dissatisfied rate was 26.67% (12/45), and the overall satisfaction rate was 73.33% (33/45); there was a significant difference in nursing satisfaction between the two groups of patients after intervention (*X*^2^ = 6.480, *P* < 0.05).

**Figure 2:** CRS-R scores of the two groups of patients ($\bar{x}$ ± *s*). Note: the abscissa represents before and after the intervention, and the ordinate represents CRS-R scores and points; the CRS-R scores of the patients in the experimental group before and after intervention were (3.54 ± 1.17) points and (20.25 ± 1.37) points, respectively; the CRS-R scores of the control group before and after intervention were (3.59 ± 1.18) points and (17.14 ± 1.26) points, respectively; there is a significant difference in the CRS-R scores of the experimental group before and after the intervention (*t* = 62.219, ^*∗*^*P* < 0.05); there is a significant difference in the CRS-R scores of patients in the control group before and after the intervention (*t* = 52.655, ^*∗*^*P* < 0.05); there is a significant difference in CRS-R scores between the two groups of patients after the intervention (*t* = 11.208, ^*∗*^*P* < 0.05).

**Figure 3:** Comparison of HAD scores between the two groups ($\bar{x}$ ± *s*). *Note.* The abscissa indicates before and after the intervention, and the ordinate indicates HAD scores and points; the HAD scores of the patients in the experimental group before and after the intervention were (35.81 ± 3.25) points and (5.36 ± 1.21) points, respectively; the HAD scores of the patients in the control group before and after the intervention were (35.88 ± 3.22) points and (13.29 ± 2.53) points, respectively; there is a significant difference in the HAD scores of the experimental group before and after the intervention (*t* = 58.901, ^*∗*^*P* < 0.05); there is a significant difference in the HAD scores of patients in the control group before and after the intervention (*t* = 37.005, ^*∗*^*P* < 0.05); there is a significant difference in the HAD scores of the two groups of patients after the intervention (*t* = 18.968, ^*∗*^*P* < 0.05).

**Table 1:** Comparison of general information of the two groups of patients.

	Experimental group (*n* = 45)	Control group (*n* = 45)	*x* ^2^/*t*	*P*
Age (year, *x* ± s)	46.75 ± 3.32	46.69 ± 3.29	0.086	>0.05
Gender [*n* (%)]			0.178	>0.05
Male	23 (51.11)	21 (46.67)		
Female	22 (48.89)	24 (53.33)		
BMI (kg/m^2^)	26.27 ± 1.59	25.89 ± 1.63	1.119	>0.05
Smoking [*n *(%)]			0.045	>0.05
Yes	20 (44.44)	21 (46.67)		
No	25 (55.56)	24 (53.33)		
Drinking [*n *(%)]			0.178	>0.05
Yes	22 (48.89)	24 (53.33)		
No	23 (51.11)	21 (46.67)		
Place of residence [*n *(%)]			0.050	>0.05
Urban	31 (68.89)	30 (66.67)		
Rural	14 (31.11)	15 (33.33)		
Type of disease [*n *(%)]				
Abdominal infection	28 (62.22)	25 (55.56)	0.413	>0.05
Respiratory tract infection	11 (24.44)	13 (28.89)	0.227	>0.05
Urinary system infection	6 (13.33)	7 (15.56)	0.089	>0.05

**Table 2:** Comparison of the nursing effect between the two groups of patients [*n* (%)].

Groups	*n*	Significantly effective	Effective	Ineffective	Total effective rate
Experimental group	45	26 (57.78)	16 (35.56)	3 (6.67)	42 (93.33)
Control group	45	21 (46.67)	10 (22.22)	14 (31.11)	31 (68.89)
*X* ^2^					8.775
*P*					<0.05

**Table 3:** Comparison of GCS scores between the two groups of patients ($\bar{x}$ ± *s*).

Groups	*n*	Limb response		Eye-opening response		Verbal response	
		Before intervention	After intervention	Before intervention	After intervention	Before intervention	After intervention
Experimental group	45	2.31 ± 0.47	4.73 ± 1.12	1.96 ± 0.24	3.51 ± 0.49	2.23 ± 0.76	4.13 ± 0.67
Control group	45	2.46 ± 0.42	3.17 ± 0.93	1.83 ± 0.37	2.18 ± 0.54	2.29 ± 0.77	3.12 ± 0.47
*t*		1.596	7.188	1.977	12.236	0.372	8.279
*P*		＞0.05	<0.05	＞0.05	<0.05	＞0.05	<0.05

## Data Availability

No data were used to support this study.
